This article has been retracted.

# Left Heart Failure Caused by Capacity Overload in Peritoneal Dialysis Patients

**DOI:** 10.1155/2022/5422333

**Published:** 2022-05-14

**Authors:** Lin Zhang, Xiaocui Zhang, Song Xue

**Affiliations:** ^1^Department of Nephrology, Municipal Hospital Affiliated to Xuzhou Medical University, Xuzhou First People's Hospital, Xuzhou, China; ^2^Department of Pediatrics, East Hospital of the Affiliated Hospital of Xuzhou Medical University, Xuzhou, China; ^3^Department of Cardiology, Affiliated Huaihai Hospital of Xuzhou Medical University, Xuzhou, China

## Abstract

**Background:**

This study sets out to investigate the incidence of acute left ventricular failure in peritoneal dialysis patients with different volume loads and to analyze the related risk factors for LVF in these patients.

**Methods:**

This study involved patients who received peritoneal dialysis in our hospital between September 2018 and January 2021. The demographic data and biochemical indicators of the patients were collected. The bioimpedance analysis method was used to determine the volume overload [overhydration (OH)] level of patients, and cardiac color Doppler ultrasound was used to detect changes in their cardiac structure. According to the LVF diagnostic criteria of symptoms and laboratory tests, the patients were divided into the LVF and non-LVF groups and then divided according to their OH level into the normal volume (OH ≤1.1 L) and volume overload (OH >1.1 L) groups. The incidence of LVF in was analyzed in patients with different volume loads, and logistic regression was used to identify the risk factors for LVF.

**Results:**

Among the 226 peritoneal dialysis patients enrolled in this study, 125 patients (55.3%) had LVF. The normal volume group (*n* = 68, 30.1%) included 22 patients (32.4%) with LVF, and the volume overload group (*n* = 158, 69.9%) included 84 patients (53.2%) with LVF. In the volume overload group, 74 patients (46.8%) had subclinical volume overload, including 35 patients (47.3%) with LVF, and 84 patients (53.2%) had clinical volume overload, including 65 patients (77.4%) LVF. Multivariate logistic regression analysis revealed a high OH level (OR = 1.862, 95% CI: 1.353–2.668, *P* < 0.001) and low hemoglobin level (OR = 0.845, 95% CI: 0.721–0.980, *P* = 0.008) to be independent risk factors for LVF.

**Conclusions:**

LVF has a high incidence in peritoneal dialysis patients, especially those with volume overload. A high OH level and low hemoglobin level are independent risk factors for LVF.

## 1. Introduction

The mortality rate of patients with chronic kidney disease (CKD) comorbid with cardiovascular disease (CVD) is 10-fold that of healthy individuals of the same age [1]. According to the dialysis transplant registration report of the Chinese Medical Association's Kidney Disease Branch, approximately 51% of patients who receive dialysis in China die from CVD and cerebrovascular disease [2, 3]. Clinical symptoms of include acute pulmonary edema, severe dyspnea, irritability, cough, cough, and pink foamy sputum [4, 5].

In CKD, volume overload is common in patients who receive peritoneal dialysis and is closely related to a poor prognosis [6]. However, to date, there have been few studies on the quantitative detection of volume load status in transperitoneal patients, or on the incidence of left heart failure (LVF) and its influencing factors in patients with different volume loads. This study aimed to assess the volume status of peritoneal dialysis patients using bioelectrical impedance analysis, examine the incidence of LVF in patients with different volume loads, and determine the risk factors for LVF, with a view to providing a basis for improving LVF prevention and treatment.

## 2. Methods

### 2.1. Patients

Patients who received regular peritoneal dialysis treatments in the Abdominal Dialysis Center of our hospital (Municipal Hospital Affiliated to Xuzhou Medical University) between September 2018 and January 2021 were enrolled. The patients were followed up for 1 year, and their data were collected. To be included, patients needed to be aged 18 years old or above and have a dialysis age of at least 3 months. The following were excluded: (I) patients with amputations; (II) patients with metal implants anywhere in their bodies; and (III) patients with local edema, such as those with deep vein thrombosis of the lower extremities. Dialysate containing glucose was used for all patients. This study was approved by the ethics committee of Municipal Hospital Affiliated to Xuzhou Medical University, and all participants signed an informed consent form.

According to the LVF diagnostic criteria of symptoms and laboratory tests, the patients were divided into an LVF group and a non-LVF group. Differences in clinical data, laboratory examination results, and the adequacy of peritoneal dialysis between the two groups were compared, and the possible risk factors for LVF were analyzed. According to the volume overhydration (OH) evaluation index, the patients were divided into two groups: the normal volume group (OH ≤1.1 L) and the volume overload group (OH >1.1 L) [7, 8]. According to the level of clinical edema, the volume overload group was divided into two subgroups: the clinical overhydration (COH) subgroup (patients with peripheral edema and/or pulmonary edema) and the subclinical overhydration (SCOH) subgroup. There are no clinically obvious signs or symptoms of edema [9]. The incidence of LVF in patients in the different volume load groups was calculated.

Initially, 236 patients were enrolled in this analysis. However, four patients who were diagnosed with deep vein thrombosis of the lower extremities were excluded, as were six patients with missing data. The final analysis included 226 patients (Figure 1).

### 2.2. Data Collection

#### 2.2.1. Demographic Data

Patient demographic data were collected, including sex, age, height, weight, dialysis age, primary disease, and comorbidities. CVD included conditions such as myocardial infarction, angina pectoris, coronary artery bypass grafting or stent implantation, congestive heart failure, stroke, transient cerebral ischemic attack, and peripheral vascular disease. Nutritional status was assessed using the subjective global assessment (SGA), and the Charlson Comorbidity Index (CCI) was used for assess the patient's comorbidities. Body mass index (BMI) is calculated using the following formula [10]: the square of weight/height of BMI = kg/m^2^. The edema level was evaluated as follows: edema below the ankle was defined as mild; edema below the knee was defined as moderate; and edema above the knee or systemic edema was defined as severe. Patients' blood pressure was measured, and the use of antihypertensive medications, including calcium channel blockers, angiotensin receptor blockers, angiotensin-converting enzyme inhibitors, receptor blockers, and diuretics, was recorded.

#### 2.2.2. Biochemical Indicator

Fasting venous blood was collected from the patients. Hemoglobin (Hb) was detected with a whole blood cell analyzer. Routine biochemical indicators, such as serum albumin (Alb), were detected using an automatic biochemical analyzer. The concentration of high-sensitivity C-reactive protein (hs-CRP) was determined using the scattering rate turbidimetric method. B-type natriuretic peptide (BNP) was detected by rapid fluorescence immunoassay.

#### 2.2.3. Peritoneal Transport Characteristics and Dialysis Adequacy

The 4-hour dialysate/plasma creatinine ratio (4hD/Pcr) was determined using a standard peritoneal balance assay, and the urea clearance index was also calculated. The residual renal function (RRF) is calculated using the following formula: RRF = {[urinary creatinine (mmol/L)/blood creatinine value (*μ*mol/L)] × urinary volume (L) × 7 + [urinary urea nitrogen (mmol/L)/blood urea nitrogen (mmol/L)] × urinary volume (L) × 7}/2.

#### 2.2.4. OH Status

A body composition analyzer was used to determine the level of OH. During measurement, the patient was instructed to remove any metal objects. The patient was told to take the supine position and keep their limbs apart relaxed. Electrode pads were then placed on the right metacarpophalangeal joint, right wrist joint, right metatarsophalangeal joint, and right ankle joint, and wires were connected for testing. The detection value was expressed as OH (L).

#### 2.2.5. LVF Diagnostic Criteria

In the dialysis patients, acute LVF is accompanied by symptoms and signs of pulmonary edema, mainly dyspnea. Rapid bedside measurement of plasma atrial natriuretic peptide (ANP) or BNP levels is necessary to distinguish pulmonary and cardiogenic dyspnea: significant increase in ANP and BNP in cardiogenic edema (BNP >80 pg/mL indicates left ventricular filling pressure elevation, which constitutes an important diagnostic basis for heart failure). Secondary heart failure is usually accompanied by significant weight gain and/or edema, as well as hypertension. Auxiliary examinations were performed using chest X-ray, electrocardiogram, and echocardiography. Echocardiography was used to measure the size of the two ventricular chambers. Ventricular diastolic function impairment was indicated by ventricular wall hypertrophy and stiffness under ultrasound. According to the above signs of laboratory examination and imaging examination, LVF was confirmed by a clinician.

### 2.3. Statistical Methods

SPSS 22.0 software (IBM Corporation, United States) was employed for statistical analysis of the data. Normally distributed measurement data were expressed as mean ± SD. The independent-samples *t*-test and Mann–Whitney *U* test were used for comparisons between groups. Count data were compared between groups using the chi-square test. Single-factor logistic regression analysis was used to screen the variables that may be potential risk factors for LVH; variables with *P* < 0.10 were incorporated into a multivariate logistic regression equation to identify independent risk factors for LVH. A two-sided test was used, and *P* < 0.05 was regarded as indicating a statistically significant difference.

## 3. Results

### 3.1. General Information of the Study Participants

This study enrolled 226 patients who received peritoneal dialysis between September 2018 and January 2021. The patients had a median age of 61.20 (48.89, 65.33) years, and the majority (126/226, 55.8%) were males. The median dialysis age was 48.77 (18.08, 72.75) months, and the median CCI score was 2.00 (2.00, 3.00). The primary disease was chronic glomerulonephritis in 98 cases (43.4%), diabetic nephropathy in 22 cases (9.7%), polycystic kidney disease in 9 cases (4.0%), and hypertensive nephrosclerosis in 4 cases (1.8%), and in 93 cases (41.2%), the cause was unknown (Table 1).

### 3.2. Incidence of LVF

Of the 226 peritoneal dialysis patients included in this study, 125 patients (55.3%) had LVF. The study participants were divided into two groups: the normal volume group (n = 68, 30.1%), which included 22 cases (32.4%) of LVF, and the volume overload group (n = 158, 69.9%), which was subdivided into the SCOH subgroup (n = 74), which included 35 cases (47.3%) of LVF, and the COH subgroup (n = 84), which included 65 cases (77.4%) of LVF.

### 3.3. Comparison of Clinical Indicators

There were no statistically significant differences between the two groups of patients in terms of age, sex ratio, dialysis age, BMI, comorbidities, diastolic blood pressure, total urea clearance index, and RRF. Compared with the non-LVF group, the LVF group showed significant increases in ACEI/ARB drug use, systolic blood pressure, BNP, 4hD/Pcr, and OH value, but their Hb level, blood Alb level, and left ventricular ejection fraction were significantly reduced; these differences were statistically significant (*P* < 0.05).

### 3.4. Risk Factors Related to LVF

The results of single-factor logistic regression analysis showed that systolic blood pressure, taking ACEI/ARB drugs, OH value, Hb, and blood Alb were risk factors LVF. After adjusting for sex, age, diabetes, CVD, systolic blood pressure, blood Alb, 4hD/Pcr factors, and multivariate logistic regression analysis revealed a high OH level [odds ratio (OR) = 1.862, 95% confidence interval (CI): 1.353–2.668, P < 0.001] and a low Hb level (OR = 0.845, 95% CI: 0.721–0.980, P = 0.008) to be independent risk factors for LVF (Table 2).

## 4. Discussion

In this study, the incidence of LVF in recipients of peritoneal dialysis was 55.3%. In the normal volume group, subclinical volume overload group, and clinical volume overload group, the incidence of LVF was 32.4%, 53.2%, and 77.4%, respectively. A high OH level and low Hb level were identified as independent risk factors for LVF in patients with CKD receiving peritoneal dialysis.

CVD is a common and serious complication in patients with CKD [11]. Patients with CKD and CVD often suffer from acute LVF due to left ventricular hypertrophy, abnormal cardiac anatomy, and volume overload factors, which manifest as acute congestion of the pulmonary circulatory system. The main manifestations of heart disease in CKD include left ventricular hypertrophy, acute and chronic heart failure, and coronary artery disease. However, LVF is the most serious pathological change and is an important risk factor for a series of cardiovascular and cerebrovascular events [4, 12]. Multiple studies have shown that LVF is an important predictor of CVD death in dialysis patients [13]. Therefore, in-depth study of the incidence of LVF and its influencing factors in the dialysis population has important clinical significance.

The incidence of LVF in this cohort of peritoneal dialysis patients reached 55.3%, which is similar to the results of Yang et al. [14]. In Wang et al.'s study [15] of 231 peritoneal dialysis patients, the incidence of cardiovascular complications was as high as 95%, which exceeded the incidence in this study. This difference in results may be related to the lower Hb level and the higher proportion of patients with CVD comorbidities in cohort. Research has found that refractory hypertension is common among peritoneal dialysis patients with volume overload and is also an independent risk factor for LVF [16, 17]. The proportion of patients with volume overload in our cohort reached 53.2%, and the prevalence of LVH in the COH group was as high as 77.4%. This observation suggests that LVF is common in peritoneal dialysis patients, especially those with volume overload. In the volume overload group, 46.8% of patients had SCOH; the incidence of LVH in this patient subgroup reached 47.3%. These findings highlight the need for clinicians to pay close attention to the evaluation of cardiac structure in peritoneal dialysis patients without obvious clinical symptoms of volume overload.

In this study, the OH value in the LVF group was significantly higher than that in the non-LVF group. Multivariate logistic regression analysis showed a high OH level to be an independent risk factor for LVF. During long-term peritoneal dialysis, the volume load of patients gradually increases with the gradual decrease of RRF. Long-term volume overload causes the proliferation and hypertrophy of cardiomyocytes, and large amounts of interstitial cell infiltration and fibroblast proliferation can be seen around the cardiomyocytes. At the same time, the activation of nerve and humoral factors can lead to cardiomyocyte hypertrophy, apoptosis, and fibrosis, eventually resulting in left ventricular hypertrophy and LVF [18]. Previous studies have found that high-frequency hemodialysis is beneficial for patients, because it can improve volume load control, thereby reducing left ventricular myocardial mass and subsequently, the mortality rate of CVD; this exemplifies the close relationship between volume overload and LVF [19].

This study found that a low Hb level is also an independent risk factor for LVF. Levin et al. [20] studied 175 patients with CKD, who had an endogenous creatinine clearance rate of 25.5 ± 17 mL/min; consistent with the results of the present study, they found that for every 10 g/L drop in Hb, the risk of CVD increased by 6%. Most patients who receive dialysis develop anemia. Some scholars have reported that left ventricular mass index and Hb are negatively correlated in peritoneal dialysis patients [21]. In anemia, the number of red blood cells decreases, which can trigger a decrease in blood viscosity. Under the synergistic effect of hypoxia, nitric oxide activity increases, vasodilatation and decreased vascular resistance cause a reduction in afterload, and decreases occur in venous return resistance, heart rate, and stroke output. The rise in blood volume elevates the circulating blood volume and causes an increase in preload, thus forming the phenomenon of “high excretion and low resistance.” In the long term, the decline in afterload and the rise in preload and left ventricular filling eventually lead to an increase in left ventricular mass, causing LFH. Studies have shown that correcting anemia in patients with CKD can partially reverse ventricular hypertrophy, thereby reducing the incidence of LVF [13, 22]. Whether anemia correction in patients receiving peritoneal dialysis can help to reverse LVF is deserving of further study.

### 4.1. Limitations

Our research has some shortcomings. First, this study is a cross-sectional study, so it is impossible to determine the causal relationship between OH, Hb, and LVF. Further prospective clinical studies are needed to confirm the results of this study. Secondly, this study evaluated clinical volume overload and subclinical volume overload based on whether the patient had peripheral edema and clinical symptoms and signs. Therefore, judgment error cannot be completely ruled out, and imaging examination results should be included in future research to reduce the risk of such error. Further, it may be more meaningful to measure the ambulatory blood pressure of patients at the same time and to analyze its relationship with LVF.

## 5. Conclusions

In summary, LVF is common in patients who receive peritoneal dialysis, especially those with volume overload. A high OH level and low Hb level are independent risk factors for LVF.

## Figures and Tables

**Figure 1:** Patient screening and enrolment. LVF, left heart failure; SCOH, subclinical overhydration; COH, clinical overhydration.

**Table 1:** Clinical data of 226 peritoneal dialysis recipients.

Variables	Value
Age (years), M (1/4, 3/4)]	61.20 (48.89, 65.33)
Male, *n (%)*	126 (55.8)
Peritoneal dialysis age (month), M (1/4, 3/4)	48.77 (18.08, 72.75)
BMI (kg/m^2^), mean ± SD	22.33 ± 2.84
*Comorbidities, n (%)*	
Diabetes	45 (19.91)
Hypertension	152 (67.26)
CVD	66 (29.20)
CCI score (points), M (1/4, 3/4)	2.0 (2.0, 3.0)
SBP (mmHg), mean ± SD	142.12 ± 16.27
DBP (mmHg), mean ± SD	86.40 ± 11.32
*Antihypertensive drug use, n (%)*	
ACEIs/ARBs	126 (55.75)
CCBs	104 (46.02)
*β*-receptor blocker	93 (41.15)
Diuretics	88 (38.94)
*Edema,n(%)*	
Mild	86 (38.05)
Moderate	12 (5.31)
Severe	3 (1.33)

BMI, body mass index; CVD, cardiovascular disease; CCI, Charlson Comorbidity Index; SBP, systolic blood pressure; DBP, diastolic blood pressure; ACEI, angiotensin-converting enzyme inhibitors; ARB, angiotensin receptor blockers; CCBs, calcium channel blockers.

**Table 2:** Logistic regression analysis of factors related to LVF in peritoneal dialysis patients.

Variable	Univariate analysis			Multivariate analysis		
	OR	95% CI	*P* value	OR	95% CI	*P* value
Male sex	1.62	0.67–3.41	0.35	2.51	0.82–5.02	0.13
Age (per 1-year increase)	1.056	0.75–1.05	0.76	1.04	0.93–1.07	0.57
BMI (1 g/m^2^ per increase)	1.46	0.92–1.59	0.12	—	—	—
Combined with diabetes	2.08	0.88–8.03	0.04	1.22	0.30–4.83	0.47
Combined with hypertension	1.06	0.47–2.45	0.84	—	—	—
Combined with CVD	1.53	0.82–3.66	0.28	1.70	0.64–5.08	0.32
ACEI/ARB use	256	1.30–6.06	0.01	2.74	0.9I–7.04	0.06
SBP (1 mmHg per increase)	1.03	1.00–1.15	0.01	1.02	0.90–1.04	0.09
Hb (1 g/L per increase)	0.95	0.97–0.99	0.01	0.97	0.94–0.98	0.01
Blood alb (1 g/L per increase)	0.85	0.81–0.99	0.03	0.97	0.84–1.12	0.44
40.01 per 4hD/Pcr (0.01 per increase)	1.03	1.00–1.07	0.06	0.99	0.96–1.03	0.99
RRF (1 mL/min per increase)	0.89	0.73–1.04	0.11	—	—	—
Volume load (1 L per increase)	1.72	1.25–2.31	<0.001	1.73	1.27–2.35	<0.001

LVF, left heart failure; OR, odds ratio; CI, confidence interval; BMI, body mass index; CVD, cardiovascular disease; alb, albumin; 4hD/Pcr, 4-hour dialysate/plasma creatinine ratio; RRF, residual renal function.

## Data Availability

No data were used to support this study.
